RETRACTED

# The Spread, Rise, and Fall of University Students' Interconnected Internet Public Opinion in the Age of Big Data

**DOI:** 10.1155/2022/9196913

**Published:** 2022-08-16

**Authors:** Meng Wang

**Affiliations:** Zhengzhou University of Aeronautics, School of Civil Aviation, Zhengzhou 450046, China

## Abstract

With the interconnected network's quick growth and widespread adoption, it has only made sense that it would serve as a hub for the dissemination of ideologies and cultural information as well as an amplifier for public opinion. The world is dualistic. The popularity of the connected network has both positive and negative effects on society. It makes people's lives more convenient, but it also has some drawbacks. Public opinion will quickly build up on the interconnected network as network communication becomes a significant method of disseminating social information, and the number of public opinion events on the interconnected network will also rise. Accurately understanding the law of higher education students' online public opinion to effectively direct and utilise online public opinion to carry out ideological education for students and to realise the establishment of students' good values, mental health, and behavioural norms, it is necessary to understand how to spread and rise and fall in the era of big data work. The parameter inversion model of online public opinion is established in this article based on the aforementioned issues. The parameter inversion algorithm is used to calculate the trend value of online public opinion, and the degree of fitting between the trend value of actual data and the trend value of parameter inversion is compared. The study discovered that the experiment's fitting value is as high as 90%. The model's prediction of the overall trend of the event development is correct, indicating that the model parameters are inverted, even though the actual public opinion data are affected by a variety of random factors, so some deviations may occur at local points. The internal law of the evolution of events that spread public opinion has been discovered, and it can be used to accurately describe the evolution and development of the public opinion dissemination process as it is driven by its internal mechanism. In the age of big data, this article analyses and summarises the rise, fall, and distribution of online public opinion among students at institutions of higher education. It also serves as a guide for monitoring and directing online public opinion in colleges and other institutions of higher education.

## 1. Introduction

Online comments and opinions made by students at higher education institutions with the aid of interconnected networks of information technology and media on certain related hot topics in real life are referred to as online public opinion. [1]. The formation of values, the growth and development of students themselves, and the interconnected network public opinion of institution of higher learning students all have significant effects on how students' work develops. The channels and methods used to publish the ontology of network public opinion are referred to as the media of network public opinion. In the big data era, information is disseminated between audiences and disseminators in a variety of interactive forms, with various network terminals serving as the primary media. The communication components and operation mechanisms of the multimedia network public opinion in the big data environment form a comprehensive whole, and they cooperate to promote the growth and evolution of the network public opinion. The fundamental building blocks of network public opinion are its communication components, and its operation mechanism is its governing law [2, 3]. The network public opinion subject is drawn to the network public opinion object through the starting mechanism, and the network public opinion media disseminate the ontology in the network public opinion space. This self-interest mechanism and polarisation mechanism are always put into action during the communication process, which completes the aggregation and diffusion of ideas. With the help of these analyses, we can gain a solid understanding of the principles and processes underlying the creation and operation of multimedia network public opinion against the backdrop of big data, allowing us to research potential solutions to control network public opinion creation and development and create a more harmonious network ecology [4].

RETRACTED

Numerous social platforms are constantly emerging as a result of the network technology's quick development, making it easier for people to communicate. The openness and virtuality of the interconnected network, however, make it impossible to effectively control people's speech when they communicate on it. Once the public opinion on this topic appears online, it could lead to severe social inconsistencies. In particular, the lack of regulations and effective oversight in the connected network is the primary cause of this phenomenon, making it a crucial forum for online users to express their emotions [5]. It can be challenging to manage online public opinion because some users of connected networks who experience difficulties or frustrations in their lives may decide to express their feelings on the connected networks. On the basis of this, it is necessary to forecast and analyse the evolution trend of the public opinion within the connected network. While university students make up the majority of the online public opinion, each student has a unique professional background, family situation, and set of morals. As a result, navigating the big data era is more challenging. When attempting to influence online public opinion, various students will exhibit a variety of attitudes, opinions, emotional responses, and behavioural patterns. Institutions of higher learning students have obvious ups and downs as their online public opinion changes in the big data era. They make up the majority of the online public opinion. Network public opinion offers new features in the subject, content, media, speed, and scope of influence in the big data era. In order to achieve effective supervision and guidance of online public opinion, reduce the negative effects of harmful online public opinion, and keep up with the times as student workers and ideological guides in colleges and institutions of higher learning, we must master the characteristics of the big data era in addition to monitoring and strengthening effect and natural attenuation law of institution of higher learning students' online public opinion.

The process by which social subjects translate their opinions on current hot topics or real focus topics from the conventional real environment to the virtual network public platform is known as the formation of network public opinion, gathering experimental social network data and choosing a model to predict public opinion. The relevant public opinion data from the actual social network is extracted and stored in the local database in this study using big data technology. The characteristics of the public opinion data are combined with the analysis and processing of the data, and useful experimental data are extracted for use as forecast input data and test data for public opinion communication models. This article presents an algorithm to complete the parameter inversion of the public opinion propagation model based on the actual social network public opinion big data and neural network after understanding some common public opinion prediction models. The parameters of actual cases are reversed based on this model. This algorithm is capable of accurately predicting both the specific public opinion heat value and the subsequent online public opinion propagation trend.

The originality of this article is as follows. This article examines the public opinion propagation law of actual social networks based on actual data, studies and analyses the hotspot discovery algorithm in the network public opinion monitoring system, and performs parameter inversion on the network public opinion propagation law based on the growing public opinion big data in order to adapt to the rapid development of interconnected network technology. For data fitting, process simulation, and trend prediction of online public opinion communication, the parameter inversion of the public opinion communication model in conjunction with public opinion big data can be used.

RETRACTED

Chapter arrangement of this article is as follows. The first chapter of this article introduces the related research of related scholars on the spread of online public opinion; the second chapter designs a network public opinion monitoring system for big data platform, which lays the foundation for the data source of this article. In the third chapter, based on the tennis public opinion monitoring system, an inversion model of network public opinion parameters is proposed, and the fitting degree of other real data is verified by experiments. The fourth chapter is the summary of the full text.

## 2. Related Work

The spread of online public opinion exhibits the characteristics of tree-like, radioactive spread, rapid spread, and repeated superposition through various channels in the age of big data due to the more colourful and diverse ways that students at higher education institutions live, learn, and work, as well as the more complex and varied information that they encounter. Data mining at that time evolved as a result of the long-term study and advancement of database technology and the advancement of artificial intelligence research [6, 7]. The database is advanced to a greater extent thanks to data mining. It is capable of more than just searching through historical data; it can also identify possible connections between data, uncover the knowledge hidden in the data, and encourage information sharing.

Bo and J. M think that public opinion refers to the subjective reflection of certain social realities and phenomena by social groups in different historical stages, and is the comprehensive expression of group consciousness, thoughts, opinions and demands [8]. Hang-Lu and Zan expanded the narrow concept of public opinion from the perspective of national decision-making. They believed that public opinion was the social objective conditions such as people's life and feelings, social productive power, and knowledge and intelligence contained in the people, which were inevitably involved in the decision-making activities of the national decision-making body, and the subjective social and political attitude of the people towards the social objective conditions and national decision-making based on their cognition, emotion, and will. In short, it is the objective social situation and the subjective will of the people, that is, social conditions and public opinion [9]. Analysis of public opinion by Wang, Xing, and Dan is the sum total of the collective emotions, wishes, attitudes, opinions, and demands held by the public in a certain historical stage and social space on public affairs matters that are related to their own vital interests or specific events that they care about, and their performance [10]. The research group believes that the leading team of online public opinion is an important force for the institution of higher learning to check online public opinion and an important guarantee for the effective development of ideological and political education for the institution of higher learning student. Therefore, colleges and institution of higher learning should set up a network public opinion supervision team linked up and down, and cultivate high-level network information administrators and high-quality campus opinion leaders to optimise their network public opinion guidance team [11]. Zong S believes that public opinion refers to the change of people around intermediary social matters, forming a social and political attitude towards state managers, which is essentially the expression of the interest relationship between people and government; interconnected network public opinion is the social and political attitude of netizens, which contains public opinions and emotions, has positive or negative influence, and will affect people's psychology and social stability. With the help of the interconnected network, thus expanding its influence [12]. Lan believes that in the era of interconnected network popularisation and development, the information of different countries, institutions, organisations, and individuals can spread rapidly through the interconnected network, causing widespread concern and even causing emergencies. In this environment, the government will face more severe challenges from the crisis of public opinion than before. How to distinguish the truth from the complex and diverse information, grasp the direction, occupy the position, and effectively manage the network public opinion of public emergencies has become one of the important issues to maintain the government's credibility and improve its ruling ability [13]. Research by Ma P, Shu X M, and Shen S F shows that the ideological and political education activities of the institution of higher learning student have both positive and negative effects. Rational use of ideological and political education methods can play a positive role, and on the contrary, it will also have a negative impact. In the era of information network, how to make full use of the advantages of network highland, strengthen the close attention and correct guidance of institution of higher learning student' network public opinion, gradually enlarge the positive aspects of network ideological and political education, and minimise the negative effects of network as much as possible is an important task and challenge faced by college ideological and political workers [14]. English X U thinks that the network is a double-edged sword. On the positive side, the institution of higher learning student' online public opinion is the display of their right to express in cyberspace, which is conducive to shaping the symbol of spiritual civilisation, establishing public discourse space, thus promoting the development and progress of social democracy, and gradually cultivating and improving the public's awareness of power and the right to speak freely. However, from the negative aspect, the comments made by institution of higher learning student in cyberspace are mixed. If those institutions of higher learning students' comments, which have great negative effects on society, cannot be properly guided and controlled in the early stage, they will easily be taken advantage of by purposeful social evil forces, forming the embarrassing situation of network anarchism, impacting the nutritional components of social harmony, splitting and destroying the overall social structure, and causing the fault of an environment-friendly society [15]. Lin, Lei, and Nie think that public opinion space refers to the situation in which people's social and political attitudes form, change, and function, and also refers to the multidimensional interaction between the subject and object of public opinion and other basic factors in the space [16]. Jin M studies the relationship between social psychological stress and public opinion from psychological stress. He believes that when people are under social and psychological pressure, they will have certain emotional reactions and physical discomfort, and they will turn into bad emotions. Bad emotions are mainly manifested in fear and anxiety. Bad emotions will directly affect people's health, related study, work, interpersonal communication, etc., and may induce psychological and mental diseases, affect people's perception, thinking, motivation to do things, cognition, and attitude, and affect people's cognition and evaluation of society. Bad transformation of social psychological pressure will distort people's social and political attitudes, resulting in bad public opinion [17].

RETRACTED

In conclusion, it is important to successfully manage the institution of higher learning students' online public opinion and develop a scientific, effective, and reasonable institution of higher learning student network in order to ensure the healthy and orderly sustainable development of college campuses and actively lead the advanced nature of institution of higher learning students' thinking. In addition to the urgent need to foster the growth of a peaceful environment in colleges and universities, this is a crucial subject that demands urgent study in ideological and political education.

## 3. Design of Network Public Opinion Monitoring System Based on Big Data Cloud Platform

### 3.1. Analysis of the Characteristics of Network Public Opinion Communication in the Era of Big Data

The need for a network public opinion monitoring method based on big data technology [18–20] has gradually emerged as a result of the expansion of interconnected network data and the inability of the traditional network public opinion monitoring method to meet those needs. Although there are numerous technologies involved in monitoring public opinion, web crawlers, information extraction from webpages, and automatic word segmentation are among the most frequently used big data technologies overall. Online public opinion has a greater impact than traditional media, permeates all spheres of society, and spans a wide spectrum. Online public opinion has gradually grown in importance as a channel for the government in the information age to hear from citizens and comprehend their viewpoints. The network's widespread influence has reached the political sphere, further altering the leaders' perspectives and ideologies.

Studying the laws of propagation and characteristics of online public opinion during times of public crisis can benefit from an analysis of the forwarding process of online public opinion. The behaviour of information spreading through a relational network in a virtual environment is actually the forwarding behaviour of online public opinion. As a result, this section also focuses on examining the relational network-based characteristics of online public opinion spreading and how they affect the shifting of the government gatekeeper's role. We should first clarify the key definitions before analysing the network public opinion sample forwarding data. In a network public opinion forwarding process, each user of the network who participates in forwarding is viewed as a node in the forwarding network, with the original network public opinion serving as the network's initial node. The term “forwarding width” describes the number of edges directly connected to a node, or the number of times a node is forwarded directly. The number of edges sharing a single forwarding path in a forwarding network is referred to as the forwarding depth. A node that directly forwards the initial network public opinion is referred to as a “direct forwarding node,” meaning that the node is directly connected to the starting node in the forwarding network. The schematic structure is shown in Figure 1.

RETRACTED

When spreading related online public opinion, Internet users are more likely to forward the original opinion directly. Netizens are, in other words, more likely to be located near the hub of the information source. It is evident that the forwarding behaviour of users on connected networks reflects the existence of two-level spreading phenomena in the process of connected network public opinion spreading. Many users of connected networks receive information from a variety of sources, not all of which are directly related to the information sources themselves. However, this information also shows how audience netizens tend to approach the centre of information sources during the process of interconnected network public opinion spreading. This function serves as a reminder to the government that when handling public crisis public opinion, it should pay attention to the authority, rigour, objectivity, and completeness of information sources, enhance the timeliness of information disclosure, and limit the spread of public crisis public opinion on the interconnected network from the source of communication. The information that netizens are exposed to is not first-hand information, but reliable information sources are urgently required in the virtual environment where the network information is chaotic and the authenticity is hard to distinguish. In order to filter bad and false information and even rumours, especially in public opinion during times of crisis, it objectively demonstrates the need for gatekeepers, and it is clear that the government is best suited to fill this position.

### 3.2. Design of Dispatching Value Module of Network Public Opinion Communication

The hot spot discovery and tracking module is the most important component of the entire system for tracking public opinion, and is a representation of the algorithms for the realisation of these two functions in the process of system requirement analysis. The two key functions of the entire system are the discovery of recent hot events and the tracking of network users' attention events. The network public opinion analysis technology has previously incorporated some data mining technology technologies and methodologies. The seamless embodiment in this case is that the network users only need to present the analysis requirements, and the system designs the technology integration method, before providing the network users with the satisfactory analysis results [21]. The system's central processing module, the hot spot discovery and tracking module, is responsible for producing the final processing output. Following information preprocessing, the webpage information is processed in the module using the classification and clustering algorithms used in data mining, which produces index data for various analysis results.

RETRACTED

In this article, for processing and analysing online public opinion data, we adopt an operating framework that can flexibly match and freely process data, and these problems have been taken into account and implemented according to such standards when the system is implemented. In the process of realising this kind of processing, a flexible system structure and data storage mode are adopted, which can customise each level of processing methods. The database describing the tasks of network users in the system is shown in Table 1.

Hierarchical task description method enables the system to use a variety of different types of algorithms to deal with a task at the same time, and this design can make the processing process execute concurrently and speed up the processing speed of the task by multithreading. The multithreading structure flow of tasks is shown in Figure 2.

In the whole process of system task processing, tasks can be divided into several levels, and the result of each level processing is the data source of the next level. The index table of processing results with only one level is shown in Table 2.

As can be seen from Table 2, the vector identifier is the serial number of the vectors in the vector library, which can uniquely identify the vectors in a library. The result category is the category number to which the vectors belong after being processed, which is the result of system analysis. The processing results with multiple levels are shown in Table 3.

Compared with the result index table with only one layer of processing, the multilayer processing result index table has more index information of each layer, and the index result may be empty. In the process of algorithm processing, a table of the processing results of the corresponding layer will be added for each layer of processing, but sometimes, this is the case. The feature selection submodule first reads the weight vectors processed by the weight vector generation module from the file, processes these weight vectors by using the selected feature selection feature extraction algorithm and corresponding parameters according to the algorithm selection in the current task, stores the processed selected vectors into the optimised weight vectors, and calculates the weight of features by the following formula:

(1) $$\begin{array}{c} H\left(c\right)=-\sum X\left(c_{i}\right)\log\;X\left(c_{i}\right). \end{array}$$

The entropy condition is shown as follows:

(2) $$\begin{array}{c} H\left(c|x\right)=-\sum X\left(c_{i}\right)\sum X\left(c_{i}|x_{i}\right)\log\;X\left(c_{i}|x_{i}\right). \end{array}$$

The greater the information gain of features and categories, the more category information contained in features. Category information is used to measure the interdependence between two signals in a message and calculate the dependence between features and categories. The feature and all kinds of information are combined as the feature weight, and the calculation formulas of feature and class information are shown in the following equations:

(3) $$\begin{array}{c} MI\left(x,c\right)=p\left(x,c\right)\log\frac{p\left(x,c\right)}{p\left(x\right)p\left(c\right)}+p\left(x,\bar{c}\right)\log\frac{p\left(x,\bar{c}\right)}{p\left(x\right)p\left(\bar{c}\right)}, \end{array}$$

(4) $$\begin{array}{c} MI\left(y,c\right)=p\left(x,c\right)\log\frac{p\left(y,c\right)}{p\left(y\right)p\left(c\right)}+p\left(x,\bar{c}\right)\log\frac{p\left(y,\bar{c}\right)}{p\left(y\right)p\left(\bar{c}\right)}. \end{array}$$

When using document frequency for feature selection, we should first calculate the document frequency of each feature word and then select all the feature words whose document frequency is higher than a certain threshold. The characteristic of low frequency does not contain useful identification information for classification, so it has no effect on the classification results. Aiming at the periodicity of the series, the analysis method of the evolution trend of interconnected network public opinion in the big data situation is judged by variance analysis, and the periodic value is calculated. The formulas for calculating the square sum of deviation between groups and the square sum of deviation within groups are shown in the following equation:

(5) $$\begin{array}{c} S_{1}=\sum_{j=1}m\left[\frac{1}{m}\sum_{i=1}^{m}\left(i,j\right)-\bar{X}\right], \end{array}$$

(6) $$\begin{array}{c} S_{2}=\sum_{i=1}\sum_{j=1}m\left[\frac{1}{m}\sum_{i=1}^{m}\left(i,j\right)-\bar{X\left(i,j\right)}\right]. \end{array}$$

For the various system algorithms, a general platform is created. According to actual needs or the needs of network users, the system can adjust to the processing demands of different algorithms and apply them at the most advantageous times. Internet public opinion based on big data analysis can allow public opinion communicators to learn more about public opinion recipients and the information cognition contained in public opinion, and can scientifically and systematically grasp the emotional responses and psychological traits of network public opinion recipients when they receive. With the help of pertinent public opinion data, it is possible to predict with accuracy how college students will spread their opinions online and increase the effectiveness of this process.

RETRACTED

## 4. Inversion of Institution of Higher Learning Network Public Opinion Parameters Based on Big Data Drive

### 4.1. Scale-free Features of Online Public Opinion Media Based on Big Data

In the age of big data, the rise and fall of time, space, and the object of public opinion are only one manifestation of the law of the development, rise, and fall of institution of higher learning students' online public opinion. It also manifests in the strength and influence of online public opinion. In the age of big data, the network public opinion of college students is accompanied by the emergence of the budding stage, brewing, fermentation, and outbreak. The greater the impact of public opinion, the more widespread its influence and the longer its duration. This study uses a scale-free network model as the medium to examine the network public opinion communication model used by colleges and other institutions of higher learning. It is referred to as a scale-free network because the connection degree of these network nodes in the network public opinion of colleges and universities has no obvious characteristic length. The network is referred to as a weighted network if each edge has the corresponding weight assigned to it; otherwise, it is referred to as an unweighted network. The nodes in the network can have various types in addition to the edge being able to be adjusted by weight. According to this model of network formation, each network user will only show up once in the network created using the forum data from the network, and the number of times a network user interacts with the same other network user will only be taken into account once at most. As a result, the value of network users can be seen in their capacity to interact with other network users. In other words, the more you converse in a forum with other network users, the more edges and higher degrees the nodes that represent the network users will have. The network is globally coupled when any two points are connected. The coupling analysis of institution of higher learning network characteristics and its scale nature is carried out, as shown in Figure 3.

The index is quite different even though the scale-free network of institution of higher learning network clustering complies with the power-law distribution, indicating that the generation and subject of institution of higher learning students' online public opinion in the big data era are more targeted, even based on the network usage habits and subject background of institution of higher learning students, and the targeted information is pushed and disseminated. The strength of online public opinion in the big data era is closely related to the hidden social contradictions that lie behind the online public opinion of institution of higher learning students, the hot spots of students' concern, and the appeal for related interests. However, the strength of online public opinion is not always directly proportional to the influence of the crowd. The intensity of online public opinion will increase as social contradictions within institution of higher learning students' viewpoints become more ferocious, and it will decrease over time as social contradictions are gradually resolved. This article counts the public opinion data in an interconnected network forum, and the trend of the daily increase of network nodes with the date is shown in Figure 4.

RETRACTED

It can be seen from Figure 4 that the number of nodes in the plate increases unevenly, except for a sudden upward trend at the tail, whose basic trend can be described as a downward trend with random fluctuations. The relationship between network clustering index and time is shown in Figure 5.

As can be seen from Figure 5, the daily average number of edges per node in the network fluctuates greatly. Although the average value in the scale-free network construction algorithm has the meaning of power exponent, it still needs a more realistic expression method.

The high growth and volume of online public opinion data complement each other in the big data environment, and the public opinion data itself exhibits characteristics of explosive transmission that are more obvious in the big data network environment. When network public opinion data are transmitted via multimedia in the big data environment, the nonlinear reading mode of the media can help the information receiver quickly read the data they are interested in. Students at higher education institutions are free to use any form of information, including images, texts, and sounds, in accordance with their individual needs, interests, task requirements, preferences, and cognitive characteristics. The instantaneous creation of a large amount of new information is also accelerated by the quick reading and use of interconnected networks, which also speed up feedback and information dissemination. Therefore, through multimedia communication, the rapid growth of online public opinion information in the big data environment can be accelerated.

RETRACTED

### 4.2. Network Public Opinion Enthusiasm Transfer Model and Analysis

Based on the actual network degree distribution parameters in the previous section, this article constructs a scale-free network with adjustable scale index and, on this basis, constructs the actual network public opinion communication model of colleges and institution of higher learning. In the era of big data, although the development process and spread of online public opinion have certain particularity, the formation, development, and end of online public opinion is a process of interaction between objective public opinion information and subjective psychological activities. At the beginning of online public opinion, it can often stimulate the institution of higher learning student' senses and stimulate students' interest in public opinion information, which lasts for a relatively long time and has a relatively strong intensity. In order to verify the reliability of the captured data, this article analyses the keyword search volume of a hot event in the time period at that time, combined with the big data platform, and obtains the hot trend charts of the first time and the second time, as shown in Figure 6.

As can be seen from Figure 6, the hot events spread and spread as quickly as volcanic eruptions in the first five days, entering the eruption stage, reaching the peak on the fifth day, and then entering the recession stage. This stage has not aroused widespread concern like the eruption stage, and the proportion of communicators has gradually decreased, but this stage is the incubation period of derivative topics, which is a relatively sensitive stage. The actual data in this stage fluctuate greatly, because there are some random factors in this stage. After the recession, the attention of netizens showed fatigue, gradually subsided, and faded out of the netizens' field of vision after a period of time. Compare the fitting degree between the trend value of real data and the trend value of parameter inversion, as shown in Figure 7.

The network parameter inversion model in this article predicts a fitting degree of about 90%, as shown in Figure 7. The actual public opinion data may deviate from some local points due to various random factors. However, the overall trend of the event's development predicted by the model is accurate, indicating that the internal law of the development of public opinion communication events can be obtained through the inversion of model parameters and that the evolution and development law of the process of public opinion communication driven by its internal mechanism can be accurately described. Once it occurs, online public opinion spreads quickly, involves a wide audience, and exerts significant influence. Among these remarks are many that are irrational and sensitive, which frequently encourage the spiralling growth of online public opinion and make it challenging to effectively control it. In the era of data, public opinion on networks now offers fresh elements in terms of subject, content, media, speed, and influence. The characteristics of the big data era, monitoring and strengthening effect, empathy effect, natural decay law of institution of higher learning students' online public opinion, human intervention, group polarisation effect, etc. are all things that we as student workers and thought leaders in colleges and universities must master. The law of dissemination and rise and fall makes it possible to effectively supervise and direct network public opinion, reduce the detrimental effects of unfavourable network public opinion on students enrolled in institutions of higher learning, and increase the beneficial effects of favourably disposed network public opinion.

RETRACTED

## 5. Conclusions

The parameter inversion of actual public opinion data has not received much attention in the past. The algorithm presented in this article completes the parameter inversion of the public opinion propagation model and is based on real-time online public opinion and a big data platform. From the growing body of public opinion big data, this algorithm can extract the fundamental rule governing the spread of public opinion. The communication components and operation mechanisms of the multimedia network public opinion in the big data environment form a comprehensive whole, and they cooperate to promote the growth and evolution of the network public opinion. The operation mechanism is the law and mechanism of network public opinion operation, and communication elements are the fundamental components of network public opinion. The subject of network public opinion is the person who contributes to network multimedia through a variety of comments. In a big data environment, there are more multimedia network public opinion subjects overall, and different groups can be classified into various categories based on the dynamics of their online public opinion behaviour. The first group is made up of online users who are not involved in online public opinion events, and the second group consists of spokespeople and subject-matter experts for governmental bodies and legal systems. The third group is the supervisory subject. They are not only active participants in online public opinion, but also the managers in charge of keeping an eye on its integrity, handling societal crises in accordance with the law, and lessening its unfavourable effects. The fourth topic is a related one or one that has interests in online public opinion events, such as parties, victims, beneficiaries, and other stakeholders. Their opinions frequently shape the evolution of online public opinion events. The network public opinion subject is drawn to the network public opinion object through the starting mechanism, and the network public opinion media disseminate the ontology in the network public opinion space. This self-interest mechanism and polarisation mechanism are always put into action during the communication process, which completes the aggregation and diffusion of ideas. Through these analyses, we can gain a thorough understanding of the principles and procedures governing the generation and operation of public opinion on multimedia networks against the backdrop of big data, allowing us to research potential solutions to control the evolution of network public opinion and create a more harmonious network ecology.

RETRACTED

As the interconnected network has grown, it has evolved into a hub for the dissemination of ideology and culture as well as an amplifier for public opinion. A growing number of people are starting to pay close attention to how online public opinion is developing, particularly how it is having an increasing impact on colleges and other institutions of higher learning. This is due to the fact that more and more students in institutions of higher education are engaging in social practices, expressing their opinions, and doing so publicly thanks to the network's interconnectedness. Online public opinions of students in institutions of higher education have also drawn more attention. There is a rare exchange of opportunities and challenges for the ideological and political education of institution of higher learning students in the interconnected network public opinion that permeates colleges and other higher education institutions. Although this article's model for the data-driven dissemination of public opinion incorporates elements of real social networks, it still has some drawbacks. The network structure in each period, such as the growth period and the outbreak period, is assumed in the data-driven public opinion dissemination research in this article to be relatively static, but the actual network is actually undergoing dynamic evolution.

## Figures and Tables

**Figure 1:** Schematic diagram of network public opinion forwarding.

**Figure 2:** Task thread structure tree.

**Figure 3:** Cluster distribution of virtual networks in colleges and institution of higher learning.

**Figure 4:** Distribution of daily increase of network nodes.

**Figure 5:** Changes of node clustering index in network.

RETRACTED

**Figure 6:** Hot spot trend chart.

**Figure 7:** Comparison of prediction results.

**Table 1:** Network user task database table.

Serial number	Mission details	Type and width	Is it missing	Primary key
1	Task ID	Int	No	Outside
2	Task-level serial number	Int	No	Inside
3	Task-level serial number	Int	No	Outside
4	Algorithm type	Int	No	Outside

**Table 2:** Processed result index table.

Serial number	Mission details	Type and width	Is it missing	Primary key
1	Result category	Int	No	Inside
2	Vector logo	Int	No	Outside

**Table 3:** Index table of multilayer processing results.

Serial number	Mission details	Type and width	Is it missing	Primary key
1	Vector logo	Int	No	Inside
2	Tier 1 result category	Int	No	Outside
3	Tier 2 result categories	Int	Yes	Outside
4	Tier 3 result categories	Int	Yes	Outside
5	—	—	—	—

## Data Availability

The data used to support the findings of this study are available from the corresponding author upon request.

## References

[1] Fan C. X., Han S. Y. (2015). Repositioning on coping strategies of college network public opinion in big Data Era. *Journal of Shaanxi Academy of Governance*.

[2] Wang Z. Q. (2016). Institution of higher learning S . The research on American students’ data protection laws and governance in the era of big data. *International and Comparative Education*.

[3] Wei H., Han C. (2018). Coping research on public opinion of the police of social media in the era of big data[J]. *Journal of Shanxi Police College*.

[4] Yangming H. U., Tao L. I. (2016). Research on the problems and countermeasures of rural public crisis management informatization in the era of big data. *Science and Technology Management Research*.

[5] Jianhua Y. U., Cao S. (2013). Research on the impacts of network public opinion on the growth of institution of higher learning students in the new period. *The Guide of Science & Education*.

[6] Chen J., Ling F., Zhang Y., You T., Liu Y., Du X. (2022). Coverage path planning of heterogeneous unmanned aerial vehicles based on ant colony system. *Swarm and Evolutionary Computation*.

[7] Cheng F., Huang Y., Tanpure B., Sawalani P., Cheng L., Liu C. (2022). Cost-aware job scheduling for cloud instances using deep reinforcement learning. *Cluster Computing*.

[8] Bo J., institution of higher learning J. M. (2017). Research on the innovation of network public opinion guiding mechanism in colleges and institution of higher learning. *Future and Development*.

[9] Hang-Lu X. U., Zan Q. (2013). Research on the network public opinion herd mentality of institution of higher learning student. *Theory Research*.

[10] Wang X., Xing Y., Dan Z. (2015). The study of network public opinion dissemination with social network analysis under the mobile environment:A case of “haze” in Sina Micro-blog. *Library and Information Service*.

RETRACTED

[11] Research Group (2012). Research on construction of monitoring, early warning and response mechanism of the network public opinion in Liaoning Province. *Journal of Liaoning Administrators College of Police and Justice*.

[12] Zong S. (2016). Research on the supervision and early warning of the security of network public opinion in Colleges and Institution of higher learning: the security of the employment of Higher Vocational institution of higher learning students. *Electronics Test*.

[13] Lan Y. (2016). Research on the governance model of network public opinion and countermeasures in emergency under the big data background. *Library & Information*.

[14] Ma Y. P., Shu X. M., Shen S. F., Song J., Li G., Liu Q. y. (2014). Study on network public opinion dissemination and coping strategies in large fire disasters. *Procedia Engineering*.

[15] Zhenglin X. U. . (2012). A restricted view on the network public opinion of the relationship between tutors and graduate students: the analysis based on the search results of the engine’s search. *Academy*.

[16] Lin P., Liu L., Nie P., Zhu X (2013). Research on network public opinion warning index system based on feature analysis of the public opinion. *Information Technology Journal*.

[17] Jin R. M. . (2017). The influence of fragmentation of network public opinion on ideological and political education of institution of higher learning students and the countermeasures. *Management & Technology of SME*.

[18] Kong J., Yang C., Xiao Y., Lin S., Ma K., Zhu Q. (2022). A graph-related high-order neural network architecture via feature aggregation enhancement for identification application of diseases and pests. *Computational Intelligence and Neuroscience*.

[19] Zeng M., Liu R., Gao M., Jiang Y. (2022). Demand forecasting for rural e-commerce logistics: a gray prediction model based on weakening buffer operator. *Mobile Information Systems*.

[20] Zhou J., Zhang D., Zhang W. (2022). Underwater image enhancement method via multi-feature prior fusion. *Applied Intelligence*.

[21] Xiao Y. F., Huang F., Zheng Y. T. (2014). Study on the contact and blocking mechanism of network public opinion and the students action. *Journal of Shenyang Institute of Engineering(Social Sciences)*.

